The article "Coal Mine Safety Evaluation Based on Machine Learning: A BP Neural Network Model" was published in 2022. Journal: Comput Intell Neurosci.

# Coal Mine Safety Evaluation Based on Machine Learning: A BP Neural Network Model

**DOI:** 10.1155/2022/5233845

**Published:** 2022-03-14

**Authors:** Guangxing Bai, Tianlong Xu

**Affiliations:** ^1^College of Safety Science and Engineering, Xian University of Science and Technology, Shaanxi, Xian 710054, China; ^2^College of Mechanical and Electrical Engineering, University of Electronic Science and Technology of China, Chengdu 611730, Sichuan, China

## Abstract

As the core of artificial intelligence, machine learning has strong application advantages in multi-criteria intelligent evaluation and decision-making. The level of sustainable development is of great significance to the safety evaluation of coal mining enterprises. BP neural network is a classical algorithm model in machine learning. In this paper, the BP neural network is applied to the sustainable development level decision-making and safety evaluation of coal mining enterprises. Based on the analysis of the evaluation method for sustainable development of coal enterprises, the evaluation index system of sustainable development of coal enterprises is established, and a multi-layer forward neural network model based on error backpropagation algorithm is constructed. Based on the system theory of man, machine, environment, and management, and taking the four single elements and the whole system in a coal mine as the research object, this paper systematically analyzes and studies the evaluation and continuous improvement of coal mine intrinsic safety. The BP neural network evaluation model is used to analyze and study the intrinsic safety of coal mines, the shortcomings of the intrinsic safety construction of coal mines are found, and then improvement measures are put forward to effectively promote the safe production of coal mines and finally realize the intrinsic safety goal of the coal mine.

## 1. Introduction

Coal will still be the main energy source for a long time. At present, the rapid growth of the economy puts forward higher requirements for the development of the coal industry [1–6]. Therefore, we must strengthen safety production and ensure the sustainable, stable, and healthy development of the coal industry. However, the coal industry is a high-risk industry. High gas and gas outburst coal mines account for about half of China's coal mines. Coal mine safety is the top priority of the whole industrial safety production work. Coal mining enterprises have the characteristics of many personnel, scattered operations, many equipment and facilities, wide distribution, bad natural conditions, many unsafe factors, complex working environments, and difficult managements. The workplace is constantly changing [7]. The risk factors of natural disasters and production accidents always affect and restrict the safe production of coal mines. On the other hand, in recent years, with the continuous changes in the internal and external environment faced by coal enterprises and the continuous deepening of the reform of large and medium-sized state-owned enterprises, the operating conditions of coal enterprises have fluctuated. On the whole, they are in the process of continuous adaptation and re-adaptation, organization and reorganization, and innovation and re-innovation [8–11]. Coal resources are nonrenewable resources. Coal mining is bound to be restricted by the remaining reserves in the mining area, and coal enterprises will face resource depletion sooner or later. Therefore, the problem of sustainable development of coal enterprises is becoming increasingly prominent. Therefore, it is very necessary to construct a coal mine safety evaluation model based on the research on the evaluation of the sustainable development level of coal enterprises.

Academic circles and decision-making departments at home and abroad have made a lot of exploration, especially in the evaluation of the sustainable development level of coal enterprises. Machine learning can be regarded as a task. The goal of this task is to let machines (computers in a broad sense) acquire human-like intelligence through learning. A neural network is a method to realize machine learning tasks. Talking about the neural networks in the field of machine learning generally refers to “neural network learning.” It is a network structure composed of many simple units. This network structure is similar to the biological nervous system, which is used to simulate the interaction between organisms and the natural environment. An artificial neural network (ANN) is an information processing system imitating human brain model [12,13]. It has good abilities of self-learning, self-adaptation, associative memory, parallel processing, and nonlinear transformation.

How to effectively curb the occurrence of major mining accidents is the biggest problem to be solved in China's coal mine production. Coal mine safety theory is put forward in this environment. The coal mine underground is a complex and changeable man-machine environmental system. This paper attempts to evaluate the sustainable development level of coal enterprises by establishing a multi-layer forward neural network model based on the error back propagation algorithm (BP algorithm). It can avoid complex mathematical derivation and ensure stable results in the case of sample defect and parameter drift, It can also effectively avoid the classical sustainable development evaluation methods, such as the analytic hierarchy process [14–16], fuzzy mathematics [17–22], and principal component analysis [23,24] and cannot avoid the role of people's experience and knowledge and the personal subjective intention of decision-makers, which is of great benefit to solve the overall decision-making planning of coal enterprises. This paper will use the system theory to take the coal mine man-machine-environment-management system as the research object, establish the coal mine intrinsic safety evaluation system and evaluation model, comprehensively construct the coal mine intrinsic safety system through the specific and in-depth analysis of various factors of man-machine-environment-management, provide the basis for coal mine safety production and management, and improve the safety production level of the coal mine industry.

## 2. BP Neural Network Model for Sustainable Development of Coal Enterprises

### 2.1. Model Building

According to the meaning of sustainable development of coal enterprises and the principle of index system design, combined with the existing achievements and the research on the specific situation of coal enterprises, an index system including 5 criteria layers and 17 specific indicators is constructed, as shown in Figure 1. According to the evaluated problems, combined with the multi-layer forward neural network model based on the error backpropagation algorithm (BP algorithm), the neural network model for sustainable development of coal enterprises is established, as shown in Figure 2.

The model is divided into two modules: the former is the normalization module, and the latter is the BP neural network (BPNN) module [25–28]. The BPNN module in the above model adopts a three-layer BP neural network, including an input layer, a hidden layer, and an output layer P. The input of a neural network is required to be in [0 and 1], so the original data of each evaluation index shall be normalized before network learning and training. The specific normalization rules are shown in Table 1. In this way, the network input value corresponding to each evaluation index in the sample can be determined by normalization.

### 2.2. Network Training and Learning

The original data are sent to the normalization module after preprocessing. The normalization module will normalize the input data according to the rules in Table *L* to obtain 17 normalized values, and then input the normalized values into the BPNN module. According to the above analysis, the number of fuzzy neurons in the input layer of the BPNN module is 17; that is, the input signals *x*_1_, *x*_2_,...,*x*_17_ correspond to 17 normalized values; the number of output neurons is 1, i.e., output *o*, which corresponds to the sustainable development level of coal enterprises. The number *k* of neurons in the hidden layer was adjusted by the learning process to 35.

The learning process of the BP neural network is also the process of network parameter correction. The network learning system adopts the method with teachers, and the correction of network parameters adopts the gradient method. It is assumed that there are *n* system sample data: $\left\{{\hat{O}}_{a},O_{a}\right\}$, *a* = 1,2, ..., n. Here, the subscript a represents the sample serial number, ${\hat{O}}_{a}$ is the sample output, and *O*_*a*_ is the actual output. x_ia_ is input variable, *i* = 1,2, ..., 17. The input variable will be assigned to the m-th neuron of the hidden layer as its input according to the following formula:

(1) $$\begin{array}{c} x_{m}^{\prime }=\sum_{i=1}^{17}w_{im}x_{ia}, \end{array}$$

where *w*_*im*_ is the weight of the input layer neuron *i* and the hidden layer neuron *m*.

The most commonly used transfer function of BP neuron is the sigmoid function:

(2) $$\begin{array}{c} f\left(x\right)=\frac{1}{1+e^{-x}}. \end{array}$$

According to the sigmoid function, it is obtained that the function of the output *O*_*m*_′ of the hidden layer neuron *m* with respect to the input *x*_*m*_′ is

(3) $$\begin{array}{c} O_{m}^{\prime }=\frac{1}{1+e_{ia}^{-x}}. \end{array}$$

Similarly, the input and output of each unit of the output layer can also be obtained, which will not be described in detail here.

Through a certain number of network training processes, it is actually to modify the network parameter to determine the most appropriate weight, so as to minimize the residual error between the actual output *O*_*a*_ and the sample output ${\hat{O}}_{a}$ obtained by forward operation according to equations (1) and (3) for all *n* sample inputs. The residual error is as follows:

(4) $$\begin{array}{c} E=\frac{1}{2}\sum_{a=1}^{n}\left(O_{a}-{\hat{O}}_{a}\right). \end{array}$$

The correction of weight and threshold is realized by the gradient method of the back propagation algorithm. t represents the time of iterative correction, and *b*_k_ and *b*_o_ represent the neuron thresholds of the hidden layer and output layer, respectively, then the parameter correction rule of the BP neural network is

(1) The connection weight from the input layer to the hidden layer is
  (5) $$\begin{array}{c} w_{ki}\left(t+1\right)=w_{ki}\left(t\right)-\eta \frac{\partial E}{\partial b_{k}}, \end{array}$$
where i = 1, 2, ..., 17; k = 1,2, ..., 35; w_*ki*_ is the connection weight from the input node xi to the hidden layer node Rk; and *η*is the learning rate.
(2) Hidden layer neuron threshold is
  (6) $$\begin{array}{c} b_{k}\left(t+1\right)=b_{k}\left(t\right)-\eta^{\prime }\frac{\partial E}{\partial w_{ki}\left(t\right)}, \end{array}$$
where k = 1,2, ..., 35 and *η*′ is the learning rate.
(3) Connection weight from hidden layer to output layer is
  (7) $$\begin{array}{c} c_{k}\left(t+1\right)=c_{k}\left(t\right)-{\eta^{\prime }}^{\prime }\frac{\partial E}{\partial c_{k}}, \end{array}$$
where k = 1,2, ..., 35; ck is the weight from the rule layer node Rk to the output layer node O; and *η*” is the learning rate.
(4) Output layer neuron threshold is
  (8) $$\begin{array}{c} b_{o}\left(t+1\right)=b_{o}\left(t\right)-{{\eta^{\prime }}^{\prime }}^{\prime }\frac{\partial E}{\partial b_{o}}, \end{array}$$
  where *η‴* is the learning rate.

After training and learning, the evaluation network can output the evaluation value to measure the level of sustainable development, which ranges from [0,1]. In order to clarify the sustainable development level of coal enterprises, the sustainable development status is divided into four levels: the first level is sustainable development, and the score range is 0.85 < *β* ≤ 1. O; the second level is primary sustainable development, and the score range is 0.70 < *β* ≤ 0.85; the third level is the transition from traditional development to sustainable development, and the score range is 0.50 < *β* ≤ 0.70; and the fourth level is traditional development, and the score range is 0 < *β* ≤ 0.50. In this way, the sustainable development level of the enterprise can be clearly obtained from the network output value. In each evaluation work, no matter whether the evaluation result is recognized by experts or not, it can be used as a new learning sample to make the BP neural network evaluation system learn and improve continuously, so as to make it make a more accurate evaluation.

## 3. Comprehensive Evaluation Model of Coal Mine Safety

This study establishes the safety evaluation index system of each element from the four elements of man, machine, environment, and management [29,30]. The construction of a coal mine safety evaluation model needs to organically combine the four elements of man, machine, environment, and management. Therefore, man, machine, environment, and management can be regarded as four primary indicators. Among the secondary indicators, human intrinsic safety indicators are divided into physical status, psychological status, safety education status, and safety technology status. Equipment safety indicators are divided into equipment reliability and production system factors. Environmental essential indicators can be divided into two categories: geological environment and working environment. The management indicators are divided into personal injury and loss, training and education, intrinsic safety management system establishment, safety measures, basic management, emergency rescue, and enterprise safety culture.

Combining the four elements organically, a coal mine safety evaluation classification model is constructed, which can be divided into four primary evaluation indexes and 14 secondary evaluation indexes, as shown in Figure 3. The scoring standard for coal mine safety evaluation in Table 2 is established with reference to the national guiding principles of intrinsic safety.

## 4. Fuzzy Evaluation of Coal Mine Safety Based on BP Neural Network

Fuzzy neural network (FNN) is a new and better system combining neural networks and fuzzy logic systems [31–33]. The system not only has the advantages of a neural network, that is, it has the function of self-organizing and adaptive learning, but also makes up for the deficiency of a neural network, that is, it can directly deal with structured knowledge, The weights without clear network meaning in the traditional neural network give the physical meaning of the rule parameters in the fuzzy system, which is convenient to use the rule parameters to study things.

### 4.1. Fuzzy Neural Network Learning Algorithm

It is assumed that *n* and *m* are the numbers of input units and hidden units, respectively. *X* = (*x*_1_, *x*_2_,…, *x*_n_) is the input layer input of the fuzzy system. After fuzzy processing of membership function, *R* = (*r*_1_, *r*_2_,…, *r*_n_) is obtained, which is the input vector of the neural network. *Z* = (*z*_1_, *z*_2_,…, *z*_n_) is the hidden layer output vector and *Y* = (*y*_1_, *y*_2_,…, *y*_n_) is the system output vector.

W_j_ = (*w*_1_, *w*_j2_,…, *w*_jn_) is the weight vector between the j-th neuron of the hidden layer and the neurons of the input layer. The weight vectors among all neurons of hidden layer and all neurons of input layer can form a weight matrix as follows:

(9) $$\begin{array}{c} w=\left[\begin{array}{c} w_{1}\\ w_{2}\\ \vdots \\ w_{m} \end{array}\right]=\left[\begin{array}{cccc} w_{11} & w_{12} & \cdots & w_{1n}\\ w_{21} & w_{22} & \cdots & w_{2n}\\ \vdots & \vdots & \; & \vdots \\ w_{m1} & w_{m2} & \cdots & w_{mn} \end{array}\right]. \end{array}$$

v_j_ = (*v*_j1_, *v*_j2_,…, *v*_jn_) is the weight vector between the j-th neuron of the hidden layer and the neurons of the output layer. The weight vectors between all the neurons of the hidden layer and all neurons of the output layer can form a weight matrix as follows:

(10) $$\begin{array}{c} v=\left[\begin{array}{c} v_{1}\\ v_{2}\\ \vdots \\ v_{m} \end{array}\right]=\left[\begin{array}{cccc} v_{11} & v_{12} & \cdots & v_{1n}\\ v_{21} & v_{22} & \cdots & v_{2n}\\ \vdots & \vdots & \; & \vdots \\ v_{m1} & v_{m2} & \cdots & v_{mn} \end{array}\right]. \end{array}$$

It is assumed that net_*j*_^*k*^ represents the net input of the j-th neuron in layer *k* andnet_*j*_^*k*^ represents the net output of the j-th neuron in layer *k*. When the BP algorithm is adopted, the input-output mapping relationship of the network is given as follows:

Input Layer
  (11) $$\begin{array}{c} \left\{\begin{array}{c} {\text{net}}_{i}^{\left(1\right)}=r_{i},\\ y_{i}^{\left(1\right)}={\text{net}}_{i}^{\left(1\right)}. \end{array}\right) \end{array}$$
Hidden Layer
  (12) $$\begin{array}{c} \left\{\begin{array}{c} {\text{net}}_{j}^{\left(2\right)}=\sum_{i=1}^{n}w_{ji}r_{i},\\ y_{j}^{\left(2\right)}=f\left({\text{net}}_{j}^{\left(2\right)}\right). \end{array}\right) \end{array}$$
Output Layer
  (13) $$\begin{array}{c} \left\{\begin{array}{c} {\text{net}}_{k}^{\left(3\right)}=\sum_{i=1}^{n}v_{kj}y_{j}^{\left(2\right)},\\ y_{k}^{\left(3\right)}={\text{net}}_{k}^{\left(3\right)}. \end{array}\right) \end{array}$$

### 4.2. Application Steps

After determining the basic structure of the training sample and model, the network training and model application are carried out according to the following steps shown in Figure 4.

## 5. Case Study

17 evaluation indexes of 8 enterprises reflecting the state of sustainable development are selected as learning samples. All samples have been normalized according to the rules in Table 1, as shown in Table 3.

The above samples are trained through the network, and the network evaluation results are obtained, as shown in Table 4. It can be seen that the network output values of enterprise 1 and enterprise 2 are between (0.85 and 1.00), enterprise 3 and enterprise 4 are between (0.70 and 0.85), enterprise 5 and enterprise 6 are between (0.50 and 0.70), and enterprise 7 and enterprise 8 are between (0.00 and 0.50). Their development levels are in sustainable development, primary sustainable development, transition from traditional development to sustainable development, and traditional development, respectively.

Based on the evaluation results of sustainable development level, the safety evaluation of enterprise 1 is now carried out. According to the intrinsic safety evaluation index system established above, data of the coal mine site are collected as shown in Table 5. Among them, the first 10 rows are the known safety assessment data of the first 10 months, the corresponding actual safety assessment value is used as the expected output as the training sample to train the BP evaluation model, and the last 2 rows are the prediction samples, representing the safety assessment data of the next 2 months.

The four elements (man, machine, environment, and management) in the coal mine and their synthesis are calculated and analyzed by using the Matlab tool and the BP neural network program. The predicted value of the personnel intrinsic safety value is (0.86–0.85). The intrinsic safety value of the equipment is (0.93, 0.95). The intrinsic safety value of environment is (0.87, 0.80). The management intrinsic safety values are (0.92, 0.93) and (0.93, 0.95). The final predicted value of coal mine intrinsic safety system is (0.93, 0.91). Therefore, it is established that the intrinsic safety degree of coal mine enterprise 1 is level I. At the same time, it also shows that the effectiveness of the neural network model applied to intrinsic safety evaluation is limited to space, and only the system intrinsic safety data is listed here as an example.

## 6. Conclusions

This paper establishes a three-layer BP neural network evaluation model to evaluate the sustainable development level of coal enterprises and obtains the sustainable development status of each enterprise. From the output layer neurons to the input layer neurons, the connection weights are corrected layer by layer, and the error back propagation correction is continuously implemented in the process of network training and learning, so as to reduce the error between the desired output and the actual output and improve the accuracy of the network response to the input mode. The evaluation results are completely consistent with the actual situation. The advantage of this method is that it avoids the subjectivity and complex mathematical derivation in the traditional evaluation methods and can still get stable and correct results in the case of missing samples and parameter drift. It will provide scientific and theoretical guidance for the scientific decision-making of sustainable development of coal enterprises and has certain research value.

Based on the sustainable development evaluation of coal mines, the establishment of intrinsically safe coal mine is the development and sublimation of the existing safety management mode and coal mine safety quality standardization. It systematizes the new concept of coal mine intrinsic safety, and the established coal mine intrinsic safety evaluation system and evaluation model are applied to the coal mine site. It can provide theoretical basis and technical support for the safety management of coal mining enterprises, effectively improve the level of coal mine safety production, eliminate hidden dangers of accidents, prevent and control accidents, standardize and improve various safety management systems, and improve the safety production situation of coal mines.

Future research will focus on two aspects: (1) optimizing the processing process of the algorithm proposed in this paper to further improve the accuracy and efficiency of the algorithm; and (2) using big data technology to analyze and process the text data recorded in the process of coal mine production and comprehensively and systematically analyze the text data of coal mines to improve the risk precontrol ability of coal mine safety production.

## Figures and Tables

**Figure 1:** Evaluation index system of sustainable development of coal enterprises.

**Figure 2:** BP neural network model.

**Figure 3:** Coal mine safety evaluation classification model.

**Figure 4:** Network training and model application steps.

**Table 1:** Normalization rules of neural network input data.

Evaluation index	Network input					
	Range	Value	Range	Value	Range	Value
Employee medical insurance rate (%)	≤10	0.1	(10, 100)	Y/100	100	1
Per capita housing area of employees (m^2^/person)	= 0	0	(0, 20)	Y/20	≥20	1
Average education level of employees	Below medium	0.3–0.5	Fairly good	0.7	Good	0.9
Enrollment rate of employees' children (%)	≤10	0.1	(10, 100)	(Y-80)/(120–80)	100	1
Reserve production ratio (%)	≤80	0.1	(80, 120)	Y/100	≥120	1
Recovery ratio (%)	≤10	0.1	(10, 100)	Y/100	100	1
Comprehensive utilization degree of resources	Below medium	0.3–0.5	Fairly good	0.7	Good	0.9
Proportion of noncoal industry (%)	≤10	0.1	(10, 100)	Y/100	100	1
Total efficiency of raw coal (t/person)	= 0	0	(0, 4)	Y/4	≥4	1
Per capita income of miners (yuan/month)	≤1000	0.1	(1000, 10000)	Y/10000	≥10000	1
Ratio of profits and taxes on funds (%)	= 0	0	(0, 20)	Y/20	≥20	1
Land reclamation rate of mining area (%)	≤10	0.1	(10, 100)	Y/100	100	1
Standard rate of noise control in mining area (%)	≤10	0.1	(10, 100)	Y/100	100	1
Standard rate of wastewater treatment in mining area (%)	≤10	0.1	(10, 100)	Y/100	100	1
Standard rate of waste gas treatment in mining area (%)	≤10	0.1	(10, 100)	Y/100	100	1
Standard rate of solid waste discharge in mining area (%)	≤10	0.1	(10, 100)	Y/100	100	1
Million ton mortality (%)	= 0	1	(0, 1)	(1-Y)/1	≥1	0

**Table 2:** Scoring standard for coal mine safety evaluation.

Safety grade	Safety classification	Evaluation score	Characterization state
1	Intrinsic safety I	[90,100)	Safe coal mine (ideal)
2	Intrinsic safety II	[80,90)	Basic safety (good)
3	Intrinsic safety III	[70,80)	Coal mine with poor safety, early warning status (general)
4	Intrinsic safety IV	[60,70)	Unsafe coal mine, medium alarm status (poor)
5	Failure to achieve intrinsic safety	[0,60)	Unsafe coal mine, heavy alarm state (bad)

**Table 3:** Network learning sample.

Evaluation index	Network learning sample (enterprises)							
	1	2	3	4	5	6	7	8
Employee medical insurance rate (%)	0.85	0.80	0.74	0.71	0.63	0.63	0.52	0.50
Per capita housing area of employees (m^2^/person)	0.90	0.90	0.81	0.78	0.75	0.80	0.73	0.74
Average education level of employees	0.90	0.90	0.80	0.70	0.80	0.60	0.40	0.60
Enrollment rate of employees' children (%)	0.88	0.96	0.85	0.89	0.88	0.78	0.79	0.94
Reserve production ratio (%)	1.00	1.00	1.00	1.00	1.00	1.00	1.00	1.00
Recovery ratio (%)	0.88	0.78	0.92	0.88	0.81	0.79	0.69	0.77
Comprehensive utilization degree of resources	0.80	0.90	0.80	0.60	0.70	0.80	0.80	0.60
Proportion of non-coal industry (%)	0.55	0.52	0.54	0.45	0.40	0.42	0.43	0.38
Total efficiency of raw coal (t/person)	0.63	0.62	0.56	0.70	0.55	0.52	0.44	0.45
Per capita income of miners (Yuan/month)	0.86	0.80	0.77	0.55	0.63	0.45	0.70	0.66
Ratio of profits and taxes on funds (%)	1.00	1.00	1.00	1.00	0.80	0.80	0.70	0.70
Land reclamation rate of mining area (%)	0.42	0.50	0.42	0.22	0.31	0.36	0.43	0.33
Standard rate of noise control in mining area (%)	0.88	0.85	0.77	0.80	0.72	0.68	0.65	0.50
Standard rate of wastewater treatment in mining area (%)	0.90	0.80	0.80	0.78	0.75	0.60	0.56	0.54
Standard rate of waste gas treatment in mining area (%)	0.88	0.86	0.77	0.78	0.72	0.88	0.89	0.91
Standard rate of solid waste discharge in mining area (%)	0.90	0.80	0.70	0.70	0.55	0.56	0.45	0.45
Million ton mortality (%)	1.00	1.00	1.00	1.00	1.00	1.00	0.95	0.94

**Table 4:** Evaluation results.

Enterprises	Network output value	Sustainable development level	
1	0.8806	First level	Sustainable development
2	0.8952	First level	Sustainable development
3	0.7277	second level	Primary sustainable development
4	0.8096	second level	Primary sustainable development
5	0.5891	Third level	Transition from traditional development to sustainable development
6	0.6122	Third level	Transition from traditional development to sustainable development
7	0.3963	Fourth level	Traditional development
8	0.2293	Fourth level	Traditional development

**Table 5:** Data of coal mine safety.

	Man	Machine	Environment	Management	Expected value	Simulated value of BP neural network
1	0.89	0.91	0.81	0.85	0.90	/
2	0.88	0.91	0.86	0.88	0.90	/
3	0.82	0.86	0.84	0.81	0.91	/
4	0.85	0.82	0.80	0.79	0.88	/
5	0.84	0.89	0.81	0.80	0.87	/
6	0.88	0.85	0.82	0.86	0.81	/
7	0.85	0.82	0.83	0.86	0.89	/
8	0.85	0.86	0.88	0.82	0.87	/
9	0.86	0.85	0.92	0.86	0.91	/
10	0.90	0.93	0.85	0.91	0.93	/
11	0.86	0.93	0.88	0.91	/	0.93
12	0.85	0.95	0.81	0.93	/	0.91

## Data Availability

The dataset can be accessed upon request.
